RETRACTED

# Risk Factors of Arteriovenous Fistula Stenosis of Patients with Maintenance Hemodialysis

**DOI:** 10.1155/2022/2968122

**Published:** 2022-11-03

**Authors:** Meiling Gao, Jing Wang

**Affiliations:** Blood Purification Center, Changzhou Second People's Hospital, Changzhou 213000, Jiangsu, China

## Abstract

**Objective:**

To investigate the risk factors of arteriovenous fistula stenosis in maintenance hemodialysis patients.

**Methods:**

A total of 80 patients with maintenance hemodialysis in our hospital from January 2017 to January 2022 were included. According to the stenosis degree of the arteriovenous fistula, patients were divided into a stenosis group (*n* = 35) and an unobstructed group (*n* = 45). Laboratory examination data, such as the demographic characteristics of patients, past medical history, the use of traditional Chinese medicine (TCM), the TCM for improving blood circulation to promote blood circulation and remove blood stasis, and cellular immune function, were collected. Multivariate Logistic regression analysis was used to analyze the influencing factors.

**Results:**

There was no significant difference in the age, sexuality, body mass index, proportion of patients with coronary heart disease, cephalic vein diameter, radial artery diameter, albumin, fibrinogen, and blood calcium levels between the two groups (*P* > 0.05). Compared with the unobstructed group, the stenosis group had higher rates of diabetes and hypertension as well as significantly higher levels of platelets, parathyroid hormone, and D-dimer (*P* < 0.05). The proportion of TCM application in the stenosis group was 28.6% (10/35), which was significantly lower than that in the unobstructed group 57.8% (26/45). The difference was statistically significant (*χ*^2^ = 6.785, *P*=0.009). The levels of CD3+ (37.5 ± 5.1% vs. 42.0 ± 4.8%), CD4+ (35.7 ± 3.2% vs. 39.6 ± 3.1%) and CD4+/CD8+ (1.4 ± 0.3 vs. 2.4 ± 1.0) in the stenosis group were significantly lower, while CD8+ level was significantly higher (26.8 ± 5.1% vs. 18.5 ± 6.2%) than that in the unobstructed group (*P* < 0.001). Logistic regression analysis indicated that the usage of TCM was an independent risk factor for arteriovenous fistula stenosis after adjustment for other factors (odds ratio [OR] 0.302; 95% confidence interval [95% CI] 0.100–0.896; *P*=0.039).

**Conclusions:**

Less use of traditional Chinese medicine for activating blood circulation and removing blood stasis and poor cellular immune function are important factors affecting the function of the arteriovenous fistula in patients with maintenance hemodialysis, which is worthy of clinical attention.

## 1. Introduction

Chronic kidney disease (CKD) refers to chronic kidney structural and functional disorders lasting for more than 3 months for various reasons, and end-stage kidney disease is a serious form of chronic kidney disease [1]. The cardiovascular risk of patients with end-stage renal disease is significantly increased, which is significantly associated with the increased risk of coronary heart disease, heart failure, and cardiovascular disease [2]. Epidemiological studies show that the prevalence of chronic kidney disease in China is 10.8%, and the annual incidence of end-stage kidney disease accounts for about 1/10,000 of the total number of patients [3]. Maintenance hemodialysis (MHD) is a vital therapeutic method of end-stage renal disease and an effective means of renal replacement therapy [4]. Maintenance hemodialysis is a therapy that uses hemodialysis technology to prolong the life span of patients with end-stage renal disease [5]. The arteriovenous fistula has the advantages of good flow, convenience, and low infection rate, which is the preferred vascular access for maintenance hemodialysis patients [6]. The occurrence of arteriovenous fistula stenosis may affect dialysis efficiency and patients' quality of life, leading to an increase in hospitalization rate and medical costs [7]. Vascular diameter, gender, electrolyte level, and other factors may be important factors causing arteriovenous fistula stenosis. For example, long-term hyperphosphatemia can lead to vascular calcification, which affects the poor vasomotor function of vessels, and makes vessels prone to stenosis or even occlusion [8]. Therefore, the factors causing arteriovenous fistula stenosis need to be actively clarified, which plays an important role in improving the survival rate and quality of life of patients with maintenance hemodialysis. The purpose of this study was to investigate the risk factors of arteriovenous fistula stenosis in patients with maintenance hemodialysis by analyzing the clinical data.

RETRACTED

## 2. Patients and Methods

### 2.1. Patients

A total of 80 maintenance hemodialysis patients in our hospital from January 2017 to January 2022 were included, including 51 males and 29 females. Inclusion criteria: (1) patients ≥18 years who met the diagnostic criteria of end-stage renal disease; (2) patients using maintenance hemodialysis as renal replacement therapy with arteriovenous fistula as vascular access; (3) patients on hemodialysis for longer than 3 months. Exclusion criteria: (1) patients with thromboembolism history; (2) patients with serious organ dysfunction such as heart, liver and kidney or serious diseases, such as malignant tumor; (3) patients with acute diseases such as infection and gastrointestinal bleeding; (4) patients who cannot cooperate with maintenance hemodialysis or have other contraindications. This study was approved by the ethics Committee of Changzhou Second People's Hospital (No. czsh1231). All patients or guardians are informed and sign consent forms.

### 2.2. Surgical Methods of Arteriovenous Fistula

All patients undergoing maintenance hemodialysis underwent wrist cephalic veno-radial artery end-to-side anastomosis. The cephalic vein was found about 3 cm above the wrist, and the venous clamp was placed at the proximal end of the cephalic vein to block the blood flow. The distal end of the cephalic vein was ligated, and the radial arterial blood flow was blocked with an arterial clamp. The proximal cephalic vein was anastomosed to the radial artery incision with a length of about 7 mm, and the skin was sutured. Most patients go through hemodialysis three times a week, and they may increase or decrease once based on their personal conditions. The time of arteriovenous fistula functionality after construction is about 6 to 8 weeks.

According to the stenosis degree of the arteriovenous fistula, it was divided into a stenosis group (*n* = 35) and an unobstructed group (*n* = 45). Arteriovenous fistula stenosis is defined as the failure of the fistula to touch the tremor, the weak or unaudible vascular murmur, the inability to meet the needs of dialysis, and the degree of vascular stenosis detected by ultrasound by more than 75%. The other group was placed in the patency group.

### 2.3. Outcome Indicators

The following indicators were used to evaluate the differences between the two groups. (1) External application of Huoxue Huayu TCM (the TCM for improving blood circulation): The external application of in the stenosis group and the unobstructed group were recorded and compared, including external application, fumigation, soaking, and wet application. (2) Cephalic vein diameter and radial artery diameter: The cephalic vein diameter and radial artery diameter of patients in the two groups were recorded by vascular color doppler examination before the creation of the arteriovenous fistula. (3) Laboratory indicators: fasting venous blood was extracted for laboratory indicators detection before the dialysis. Platelet count was measured by an automatic blood cell analyzer. Albumin and blood calcium levels were measured by an automatic biochemical analyzer. The levels of fibrinogen and D-dimer were determined by photoelectric colorimetry. The level of parathyroid hormone (PTH) was detected by chemiluminescence. (4) Cellular immune function: the level of CD3+T lymphocytes, CD4+T lymphocytes, and CD8+T lymphocytes was detected by flow cytometry (EPICSXL, Beckman Coulter, USA), and CD4+/CD8+ was calculated.

RETRACTED

### 2.4. Statistical Analysis

Statistical analysis was performed by IBM SPSS 21.0 software. The classified variables were expressed as *N* (%), and the chi-square test was used to compare the differences between the stenosis group and the unobstructed group. Continuous variables were expressed as mean ± standard deviation, and *t*-test was used to compare the difference between the stenosis group and the unobstructed group. Multivariate logistic regression was used to analyze the risk factors of arteriovenous fistula stenosis. Bilateral *P* < 0.05 was considered statistically significant.

## 3. Results

### 3.1. Clinical Characteristics and General Data of the Patients

As shown in Table 1, a total of 80 maintenance hemodialysis patients were enrolled in this study. There were no significant differences in age, sex, body mass index, proportion of patients with coronary heart disease, cephalic vein diameter, radial artery diameter, albumin, fibrinogen, and blood calcium levels between both groups (*P* > 0.05).

### 3.2. Differences in the Use of TCM

As shown in Table 2, the proportion of TCM usage was 28.6% (10/35) in the stenosis group and 57.8% (26/45) in the unobstructed group. The proportion of TCM usage in stenosis group was significantly lower than that in the unobstructed group, with statistical significance (*χ*^2^ = 6.785, *P*=0.009).

### 3.3. Cellular Immune Function

Compared with the unobstructed group, the levels of CD3+ (37.5 ± 5.1% vs. 42.0 ± 4.8%), CD4+ (35.7 ± 3.2% vs. 39.6 ± 3.1%) and CD4+/CD8+ (1.4 ± 0.3 vs. 2.4 ± 1.0) were lower in the stenosis group. The difference was statistically significant (*P* < 0.001). The CD8+ level in the stenosis group was significantly higher than that in the patency group (26.8 ± 5.1% vs. 18.5 ± 6.2%, *P* < 0.001). See Table 3 for details.

### 3.4. Risk Factors of Arteriovenous Fistula Stenosis Were Analyzed by Logistic Regression

In Table 4 univariate analysis, the function of arteriovenous internal fistula was taken as the dependent variable (assignment: unobstructed = 0, stenosis = 1), and the use of TCM was taken as the independent variable (assignment: no use = 0, use = 1). The use of TCM was significantly correlated with the lower risk of arteriovenous internal fistula stenosis (OR 0.292; 95% CI, 0.114 to 0.750; *P*=0.011). In model 1, the OR value was 0.295 after adjusting for age, sexual and body mass index (95% CI 0.113–0.768; *P*=0.012). Based on model 1, the OR value of model 2 was 0.296 after adjusting for diabetes, hypertension, coronary heart disease, cephalic vein diameter, and radial artery diameter (95% CI 0.102–0.860; *P*=0.025). Based on model 2, model 3 adjusted platelet, albumin, serum calcium, fibrinogen, D-dimer, and parathyroid hormone, and found that the use of TCM was an independent factor in less stenosis of the arteriovenous fistula (OR 0.302; 95% CI, 0.100 to 0.896; *P*=0.039).

RETRACTED

## 4. Discussion

This study found that patients with arteriovenous fistula stenosis had higher rates of diabetes and hypertension, and higher levels of platelets, parathyroid hormone, and D-dimer. They had lower levels of CD3+, CD4+, and CD4+/CD8+, and higher levels of CD8+. It is worth noting that the application of Huoxue Huayu Traditional Chinese medicine is an independent factor affecting the occurrence of arteriovenous fistula stenosis.

End-stage renal disease is an important social and economic burden in China, and the emergence of maintenance hemodialysis has played an important role in improving the prognosis of patients with end-stage renal disease and prolonging their life expectancy [9]. Arteriovenous fistula provides sufficient blood volume for hemodialysis and is an ideal vascular access for patients undergoing maintenance hemodialysis with a long duration and few complications [10]. Factors such as radial artery diameter, blood pressure, heart rate, weight, and blood hypercoagulability state are the key factors affecting the function of the arteriovenous fistula [11]. However, the occurrence of arteriovenous fistula stenosis may affect the efficiency of hemodialysis and the quality of life of patients and is an important cause of dialysis interruption or dialysis failure [12]. Therefore, improving the factors causing arteriovenous fistula stenosis will help improve the survival rate and quality of life of patients with maintenance hemodialysis.

Previous studies have shown that age, combined hypertension, diabetes, and hypoalbuminemia are the key factors causing arteriovenous fistula stenosis [8].

The study also found a higher proportion of patients with diabetes and hypertension in the stenosis group than in the unobstructed group. Elderly patients complicated with diabetes and hypertension are prone to vascular endothelial function impairment, high blood coagulation and are easily affected b arteriovenous fistula stenosis and thrombosis. Similar to the results of this study, other studies have found that increased plasma parathyroid hormone levels significantly increase the risk of arteriovenous fistula dysfunction [13]. In recent years, some scholars have proposed that neutrophil/lymphocyte ratio and platelet/lymphocyte ratio may be important factors in predicting arteriovenous fistula stenosis [14, 15].

This study found that less use of Huoxue Huayu TCM was independently associated with the occurrence of arteriovenous fistula stenosis after adjustment for other factors (OR 0.302; 95% CI, 0.100 to 0.896; *P*=0.039). This kind of Chinese medicine has the effect of promoting blood circulation, removing blood stasis, and relieving pain. External application of traditional Chinese medicine for promoting blood circulation and removing stasis in arteriovenous fistula can not only improve subcutaneous hematoma and promote the dissipation and absorption of hematoma but also prevent the occurrence of stenosis and occlusion of arteriovenous fistula. Studies have suggested that T lymphocyte subsets may change significantly in patients with end-stage renal disease, with significantly reduced levels of CD3+, CD4+, and CD8+T lymphocytes [16]. The results of this study suggest that the levels of CD3+, CD4+, and CD8+T lymphocytes also play an important role in the occurrence and development of arteriovenous fistula stenosis. In addition to lymphocytes, a 2021 study suggested that neutrophil/lymphocyte ratio and neutrophil elastase were independent risk factors for arteriovenous fistula stenosis [17].

RETRACTED

It should be noted that this study has the following limitations. The sample size of this study was small and the study duration was short. In the future, large samples and long-term follow-up studies are needed to further verify the role of TCM for promoting blood circulation and removing stasis and cellular immune function in arteriovenous fistula stenosis in patients with maintenance hemodialysis.

## 5. Conclusion

In conclusion, in addition to age, complicated diabetes and hypertension, less use of traditional Chinese medicine and poor cellular immune function are important factors affecting the function of the arteriovenous fistula, which deserve clinical attention.

## Figures and Tables

**Table 1:** Comparison of clinical features and general data between the two groups.

	Stenosis group	Unobstructed group	*t*/*χ*^2^	*P*
*N*	35	45	—	—
Age years	53.5 ± 5.0	52.3 ± 5.2	1.071	0.287
Male *n* (%)	24 (68.6)	27 (60.0)	0.626	0.429
Body mass index (kg/m^2^)	23.3 ± 3.3	24.0 ± 4.8	−0.698	0.487
Diabetes mellitus *n* (%)	16 (45.7)	11 (24.4)	3.983	0.046
Hypertension *n* (%)	19 (54.3)	14 (31.1)	4.363	0.037
Coronary heart disease *n* (%)	12 (34.3)	9 (20.0)	2.075	0.150
Cephalic vein diameter (cm)	2.30 ± 0.31	2.36 ± 0.27	−0.937	0.352
Radial artery diameter (cm)	2.10 ± 0.23	2.18 ± 0.25	−1.329	0.188
Platelets 10^9^/L	215 ± 43	188 ± 37	2.994	0.004
Albumin (g/L)	33.4 ± 5.2	34.2 ± 4.8	−0.779	0.438
Blood calcium (mmol/L)	2.16 ± 0.22	2.23 ± 0.20	−1.282	0.204
Fibrinogen (g/L)	3.9 ± 1.8	4.1 ± 0.7	−1.431	0.157
D dimer (mg/L)	3.0 ± 0.8	2.6 ± 0.8	2.043	0.044
Parathyroid hormone (ng/L)	476 ± 124	410 ± 108	2.534	0.013

RETRACTED

**Table 2:** Comparison of TCM usage between the two groups (*n* (%)).

	Stenosis group	Unobstructed group
Used	10 (28.6)	26 (57.8)
Un-used	25 (71.4)	19 (42.2)
*χ * ^2^	6.785	
*P*	0.009	

**Table 3:** Comparison of immune function between the two groups.

	Stenosis group	Unobstructed group	*t*	*P*
CD3^+^ (%)	37.5 ± 5.1	42.0 ± 4.8	−4.030	<0.001
CD4^+^ (%)	35.7 ± 3.2	39.6 ± 3.1	−5.459	<0.001
CD8^+^ (%)	26.8 ± 5.1	18.5 ± 6.2	6.443	<0.001
CD4^+^/CD8^+^	1.4 ± 0.3	2.4 ± 1.0	−5.968	<0.001

**Table 4:** Logistic regression analysis of the use of traditional Chinese medicine in patients of the two groups on arteriovenous fistula stenosis.

	B	SE	Wald *χ*^2^	OR	95% CI	*P*
Univariate analysis	−1.230	0.481	6.546	0.292	0.114–0.750	0.011
Model 1	−1.222	0.489	6.253	0.295	0.113–0.768	0.012
Model 2	−1.217	0.544	5.009	0.296	0.102–0.860	0.025
Model 3	−1.209	0.562	4.895	0.302	0.100–0.896	0.039

Model I adjusted for age, sexual and body mass index; model 2 based on model 1, the diameter of diabetes mellitus, hypertension, coronary heart disease, cephalic vein, and radial artery were corrected; in model 3, platelet, albumin, serum calcium, fibrinogen, D-dimer, and parathyroid hormone were adjusted based on model 2.

## Data Availability

The data used to support the findings of this study are available from the corresponding author upon request.
